# Clinical Practice Pattern of Korean Medicine Doctors in Idiopathic Short Stature Treatment: A Survey Study

**DOI:** 10.1155/2022/1505643

**Published:** 2022-08-10

**Authors:** Soobin Jang, Boram Lee

**Affiliations:** ^1^Department of Preventive Medicine, College of Korean Medicine, Daegu Haany University, 1 Haanydaero, Gyeongsan-si, Gyeongsangbuk-do 38610, Republic of Korea; ^2^KM Science Research Division, Korea Institute of Oriental Medicine, 1672 Yuseong-daero, Yuseong-gu, Daejeon 34054, Republic of Korea

## Abstract

**Background:**

Korean medicine (KM) interventions are attractive for children with idiopathic short stature (ISS). We investigated the real-world clinical practice patterns of KM doctors in ISS treatment.

**Methods:**

The survey targeted KM doctors who have treated patients with ISS in KM clinical settings for >3 years. We included questions on the diagnosis and treatment patterns, effects, cost, and opinions of doctors on KM treatment for ISS. A frequency analysis was performed.

**Results:**

There were 58 respondents, and “heights of parents” (*n* = 57, 98.3%), “height, weight, and growth rate of child” (*n* = 55, 94.8%), and “amount of meals, digestive function” (*n* = 52, 89.7%) were frequently used as indicators for diagnosis and treatment. The most frequently used KM interventions were “herbal medicine” (*n* = 58, 100%), “acupuncture” (*n* = 49, 84.5%), “moxibustion” (*n* = 38, 65.5%), “dry cupping” (*n* = 26, 44.8%), and “physiotherapy” (*n* = 22, 37.9%). Herbal medicines were generally prescribed to tonify the spleen or kidney, and the most frequently used individual herbs were *Acanthopanacis cortex*, *Astragali Radix*, and *Cervi parvum cornu*. The most common acupuncture points were ST36, GB34, SP6, EX-LE5, and LI4.

**Conclusions:**

This study showed the use of KM for ISS in real-world clinical settings. In the future, well-designed clinical studies to verify the effect of KM treatment on ISS based on real-world clinical practice patterns should be actively performed.

## 1. Introduction

Idiopathic short stature (ISS) is defined as when the individual's height is two standard deviations or more below the corresponding average height for a given age, sex, and population group, in the absence of any systemic, endocrine, nutritional, or chromosomal abnormality [1]. Approximately 80% of children with short stature are estimated to have ISS [2] and its prevalence is estimated of 16 per 1,000 children [3]. In conventional medicine, recombinant human growth hormone (GH) has been used as the primary standard therapy for ISS since it was approved by the US Food and Drug Administration in 2003 [4]. However, this treatment is rather inconvenient and expensive because it requires daily parenteral administration. Additionally, concerns have been raised regarding the safety of long-term GH treatment, including a decreased sensitivity to insulin, an increased risk of type 2 diabetes, and an adverse effect on peak bone mineralization [5–7].

In South Korea, Korean medicine (KM) treatments, including acupuncture, moxibustion, and herbal medicine, also known as East Asian traditional medicine (EATM), one of the most well-known types of complementary and integrative medicine, have been widely used as an alternative treatment method to support child growth. According to a retrospective study in 2016, growth retardation was the chief complaint among children and adolescents who visited the department of Korean Pediatrics in a KM Hospital [8]. Several preclinical and clinical studies have shown that EATM therapies are effective in treating ISS [9–12]. However, clinical practice guidelines of KM for pediatric growth disorder have not been published. Therefore, an in-depth investigation of the diagnosis and treatment patterns of KM doctors (KMDs), as well as the treatment cost for ISS, may enhance the understanding of the actual healthcare situation and contribute to research that reflects real-world clinical settings.

## 2. Methods

### 2.1. Study Aim, Design, and Setting

The aim of this study was to investigate the clinical practice patterns of KMDs in ISS treatment and their therapeutic effects and costs in real-world clinical settings.

This study used a cross-sectional survey design to assess the clinical practice patterns of KMD for ISS treatment in South Korea. The survey was conducted by Mediresearch (https://www.mediresearch.co.kr), which is a professional survey research company. The company sent a questionnaire survey *via* mobile phone to KMDs affiliated with KM clinics or hospitals, based on the cooperation of the Association of Pediatrics of KM. The company recruited participants with consideration of the ratio between specialists in pediatrics and general KM practitioners. The participants were enrolled voluntarily and they were informed that responses were required for all our questions in the questionnaire. The survey was conducted anonymously between November 24 and December 23, 2020.

### 2.2. Participants

The purpose of this study was to observe the clinical practice patterns of KMD in real-world settings, not to verify the treatment effect; therefore, there was no special method for determining the sample size. We determined the minimum number of respondents as 40, with additional recruitment ongoing until the end of the study period. The inclusion criterion was >3 years of experience of ISS treatment in KM clinical settings.

### 2.3. Questionnaire

The questionnaire was developed by three traditional KM experts who discussed and selected investigation items. The experts sought to create a concise and easily readable questionnaire to raise the response rate. They conducted a pilot test with a draft questionnaire and feedback was collected. The final version of the questionnaire was developed for respondent convenience using smartphones.

The questionnaire consisted of five categories. Variable descriptions are as follows:

1. Basic demographic and clinical characteristics of KMD respondents: sex, age, duration of clinical experience, type of KMD license, working institution, monthly number of patients with ISS, and mean age group of patients with ISS.
2. Diagnosis patterns: indicators used in the diagnosis and treatment of ISS and comorbidities that are checked during ISS diagnosis and treatment.
3. Treatment patterns: which KM intervention apply, including herbal medicine, acupuncture, moxibustion, dry cupping, physiotherapy, electroacupuncture, pharmacopuncture, and chuna. Administration duration; frequency of each intervention (except herbal medicine); purpose of herbal prescription; and frequently used individual herbs and acupoint.
4. Effectiveness and cost: mean height growth (cm) before and after KM treatment, according to sex and age, and cost of each intervention.
5. Opinions on KM treatment for ISS: Korean-Western medicine collaborations for the treatment of growth disorders; essential KM interventions that should be included in health promotion program for children's growth; limitations of KM treatment for children's growth; and the appropriate herbal medicine for insurance.

### 2.4. Statistical Analyses

Frequency analysis was conducted for each question, and the ranking was confirmed by indicating the number of responses (*n*) and percentage (%). Microsoft Excel 2016 (Microsoft Corporation, Redmond, WA, USA) was used for all analyses.

### 2.5. Ethical Considerations

The study was explained to all participants prior to the initiation of the survey. Only those who voluntarily agreed to participate and for their collected data to be published were enrolled in the study. This study was approved by the Institutional Review Board of Korea Institution of Oriental Medicine (IRB No. I-2010-008-002-01).

## 3. Results

### 3.1. Basic Demographic and Clinical Characteristics of Respondents

Fifty-eight KMDs, consisting of 31 (53.4%) men and 27 (46.6%) women, participated in this study. Most respondents were aged between 30 and 49 years (86.2%). In addition, most of their clinical experience was evenly distributed between 5 and 30 years (94.8%). The average monthly number of ISS patients was “<10” (*n* = 27, 46.6%), followed by “≥10 and <30” (*n* = 17, 29.3%). The most frequent average age of ISS patients was prepubertal (≥6 and <10; *n* = 28, 48.3%), followed by preschool (≥3 and <6; *n* = 19, 32.8%) (Table 1).

### 3.2. Diagnosis Patterns of ISS in Korean Medicine

The most common indices that were referred to when diagnosing ISS were “heights of parents” (*n* = 57, 98.3%), ‘height, weight, and growth rate of child' (*n* = 55, 94.8%), and “amount of meal, digestive function” (*n* = 52, 89.7%), followed by “pattern identification” (*n* = 38, 65.5%), “growth plate test (*X*-ray)” (*n* = 37, 63.8%), “pulse diagnosis” (*n* = 36, 62.1%), “abdominal diagnosis” (*n* = 34, 58.6%), and “tongue diagnosis” (*n* = 30, 51.7%). The top comorbidity that was assessed for when diagnosing and treating ISS was “digestive diseases” (*n* = 53, 91.4%), followed by “respiratory diseases” (*n* = 33, 56.9%), and “allergic diseases” (*n* = 23, 39.7%) (Table 2).

### 3.3. Treatment Patterns of ISS in Korean Medicine

All KMDs responded that they used “herbal medicine” (*n* = 58, 100%) as an intervention in ISS treatment, followed by “acupuncture” (*n* = 49, 84.5%), “moxibustion” (*n* = 38, 65.5%), “dry cupping” (*n* = 26, 44.8%), and “physiotherapy” (*n* = 22, 37.9%). “Electroacupuncture,” “pharmacopuncture,” and “chuna” were each selected by 20 respondents (34.5%). The herbal medicine administration period typically ranged from 1 to 6 month: “≥1 and <2 months” (*n* = 12, 20.7%); “≥2 and <3 months” (*n* = 20, 34.5%); and “≥3 and <6 months” (*n* = 17, 27.6%). The frequency of other interventions was generally “once a week” in a clinical setting (Table 3).

The purpose of prescribing herbal medicines were as follows: 51.7% (*n* = 30) for “tonifying the spleen,” 19.0% (*n* = 11) for “tonifying the spleen and the kidney,” 12.1% (*n* = 7) for “tonifying the kidney,” and 10.3% (*n* = 6) for “tonifying the liver and the kidney.” The frequently used herbs for ISS treatment were “*Acanthopanacis cortex*” (*n* = 23, 41.8%), “*Astragali Radix*” (*n* = 23, 41.8%), “*Cervi parvum cornu*” (*n* = 21, 38.2%), and “*Rehmanniae Radix preparata*” (*n* = 18, 32.7%). The most frequently used acupuncture points for ISS treatment were “ST36 (Zusanli)” (*n* = 48, 82.8%), “GB34 (Yanglingquan)” (*n* = 36, 62.1%), “SP6 (Sanyinjiao)” (*n* = 32, 55.2%), “EX-LE5 (Xiyan)” (*n* = 28, 48.3%), and “LI4 (Hegu)” (*n* = 26, 44.8%) (Table 4).

### 3.4. Effectiveness and Cost of Korean Medicine Treatment for ISS

According to the response of KMDs, the mean (standard deviation) of growth height after KM treatment was 6.03 (0.98) cm before puberty and 9.03 (1.56) cm during puberty in boys; and 5.83 (1.05) cm before puberty and 8.36 (1.71) cm during puberty in girls (Table 5).

The distribution of the cost of each intervention is described in Table 6. The cost of moxibustion, dry cupping, and physiotherapy was typically <9 dollars per visit, and acupuncture was <11 dollars per visit. The cost of herbal medicine for the majority of respondents (*n* = 45, 77.6%) ranged from 156 to 268 dollars per 15 days. The daily cost of herbal medicine was between 10.4 and 17.9 dollars.

### 3.5. Opinions on the Use of Korean Medicine in ISS Treatment

Twenty-eight KMDs (48.3%) responded that ‘KM treatment is more cost-effective than GH.' By contrast, 22 KMDs (37.9%) responded that ‘It is best to combine herbal medicine, acupuncture, and GH.' Herbal medicine (decoction) was selected the most (*n* = 45, 77.6%) as an essential KM intervention that should be included in a health promotion program for pediatric growth disorders. The top herbal medicines requiring cover by health insurance for ISS treatment were Yukmijihwang-tang (*n* = 25, 43.1%), Sogunjung-tang (*n* = 14, 24.1%), Yukgunja-tang (*n* = 8, 13.8%), Sipjeondaebo-tang (*n* = 5, 8.6%), and Sagunja-tang (*n* = 3, 5.2%) (Table 7).

## 4. Discussion

This survey investigated the clinical practice patterns of KM treatment for ISS, including a detailed evaluation of diagnosis, treatment, effectiveness, and costs. Furthermore, we sought the opinions of KMDs regarding their use of these treatments. We have also previously reported a network meta-analysis [13] and an observational case series [14] of integrative KM treatment for ISS. The findings suggested that EATM plus GH might have a synergistic effect in comparison with EATM or GH alone [13]. In addition, the changes in growth indicators in children with ISS before and after KM treatment showed the potential of KM for the management of ISS [14]. However, detailed information regarding interventions and costs could not be obtained by both studies because they were secondary research studies using existing data. Therefore, we designed this survey to obtain specific information regarding ISS treatment.

Pattern identification based on KM theory could be a significant method for treating ISS because it is a primary growth disorder with an unknown cause. ISS is typically regarded as a problem with digestive disorders or lack of nourishment in KM [15]. This is consistent with the majority of respondents focusing on “tonifying the spleen (補脾) or the kidney (補腎)” as the purpose of ISS treatment in our study. In EATM, “tonifying the spleen” is defined as a therapeutic method to treat diminished functional activities of the spleen by using tonifying medicines. “Tonifying the kidney” is a general term for treating deficiency patterns/syndromes of the kidney with tonifying medicines [16].

Taken together, these data show that herbal medicine is regarded as an essential ISS treatment intervention. Furthermore, acupuncture and moxibustion are also necessary for ISS treatment. The administration period for herbal medicines was between 2 and 6 months, and the frequency of other interventions was once a week. Yukmijihwang-tang (六味地黃湯) [17], the most common herbal prescription requiring coverage by health insurance, is a representative herbal medicine for tonifying the kidney. Sogeonjung-tang (小建中湯) [18] and Yukgunja-tang (六君子湯) [19], which were the second and third most commonly recorded, are herbal medicines used to tonify the spleen. In particular, Sogeonjung-tang is a first-line KM treatment for children with a lack of appetite or poor digestion [18].

The most frequently used individual herbs for ISS treatment in clinical settings were *Acanthopanacis cortex* (五加皮), followed by *Astragali Radix* (黃芪) and *Cervi parvum cornu* (鹿茸). The effects of a complex herbal mixture containing *Acanthopanacis cortex*, *Astragali Radix*, and *Dipsaci Radix* (續斷) on height growth have been studied previously and the study showed that height gain was significantly higher in the herbal mixture group than in the placebo group after 24 weeks [12]. Additionally, *Cervi parvum cornu* is the most popular supplement for growth promotion and continues to grow in popularity [20]. In addition, ST36 (Zusanli), the acupuncture point that KMDs reported using most frequently, is actively used in traditional Chinese medicine clinical research, and its positive effect on growth has been studied [21].

All the acupoints frequently used for the treatment of ISS, except GV20 (Baihui) and CV12 (Zhongwan), were located below the knee to the toes (Table 4). This could stimulate height growth by stimulating the bones of the knee, tibia, and ankle. ST36 (Zusanli) is the most frequently selected acupoint and has been also used for the treatment of short stature in other studies [22, 23]. SP6 (Sanyinjiao)is an acupoint where the three yin meridians of the liver, spleen, and kidney meet, and is used to tonify the liver, spleen, and kidney. GV20 (Baihui) is placed at the top of the head where all yang-qi gathers, and CV12 (Zhongwan), which strengthens digestive functions, is placed at the middle of the umbilicus and the xiphisternal joint.

Several studies have conducted the economic evaluation of GH treatment on ISS [24, 25]. Furthermore, clinical trials have examined the growth effects of herbal medicines in China [26, 27]; however, studies conducting economic evaluation of complementary therapies, such as herbal medicines and acupuncture, for ISS treatment have not been published. We sought to calculate the incremental cost-effectiveness ratio of KM intervention for ISS by extracting the data from systematic reviews, randomized controlled trials, or national secondary data; however, no proper data provided the costs and growth effects of KM interventions.

Accordingly, we collected costs and height growth data in this survey, although it was not sufficient to make any conclusions. Nonetheless, we estimated that three months (the most responsive treatment period) of treatment with herbal medicine, acupuncture, and moxibustion would cost in the range of USD 1,554–1,824. The frequency and cost of acupuncture and moxibustion were assumed to be as once a week and USD 9 per session, respectively. The difference in height growth before and after KM treatment was 1.93 cm (before puberty) and 2.53 cm (puberty) in boys; and 1.69 cm (before puberty) and 2.22 cm (puberty) in girls (Table 5). Therefore, considering the relatively low cost and the effect of height growth of the KM treatment, KM treatment may be cost-effective for ISS treatment. Additionally, almost half of the KMDs who participated in this survey answered that KM treatment was more cost-effective than GH (Table 7). However, the estimated effectiveness and cost of KM treatment were based on the response of a small number of KMDs and not the actual patient data; thus, it was difficult to compare it with GH treatment (currently used treatment). In addition, as comparison with the untreated control group is impossible due to the nature of the data, the difference in growth rate before and after KM treatment reported by KMDs may not be attributed to the effect of KM treatment. Furthermore, there may be recall errors, and caution is required in interpretation. A study on the effect of KM treatment on the final adult height should be performed to evaluate the cost-effectiveness of KM treatment compared with height monitoring or GH treatment for ISS.

Currently, KM interventions for ISS are not covered by health insurance in South Korea. This is reported as the primary limitation of KM treatment for growth disorders. Several health promotion programs have reported using KM interventions for child growth in public health centers [28]. Health promotion, in contrast to clinical treatment, consists of exercise, education, herbal medicine, and acupuncture. In addition, we are developing a KM health promotion program for children's growth based on the results of this survey. Many KMDs responded that herbal medicine with a type of decoction should be included in a health promotion program; however, it is difficult to provide decoctions because of costs and quality control. Health promotion programs are generally provided free of charge to residents in need; therefore, this could help children with ISS safely and effectively.

There are several limitations in this study. First, the number of participants was small and not representative of the entire KMD population. This survey aimed to recruit KMDs who focused on pediatric care with >3 years of clinical experience with ISS rather than more respondents to investigate clinical patterns in detail. The total number of KMDs is approximately 22,000, and there are only about 130 pediatric specialists focusing on KM in South Korea [29]. In addition, the sample size was small for realistic reasons, such as the study period and funding size. Second, recall bias is likely because the survey depended on the memory of respondents. A future chart analysis study is recommended to extract more accurate data. Additionally, the cost of herbal medicines varies significantly depending on the herb; therefore, the cost effectiveness can only be assessed as reference. Nevertheless, to the best of our knowledge, this study is the first to assess the clinical treatment pattern of ISS in a real-world KM setting.

## 5. Conclusions

This study analyzed the current KM clinical practice for the treatment of ISS, focusing on diagnosis indices and treatment patterns. The effects and costs of height growth and opinions of KMDs were also investigated. In the future, studies evaluating the efficacy and cost-effectiveness of KM treatment for ISS should be performed based on real-world clinical practice.

## Figures and Tables

**Table 1:** Basic demographic and clinical characteristics of respondents.

Basic information		*n* (%)
Sex	Men	31 (53.4)
	Women	27 (46.6)

Age (years)	<30	1 (1.7)
	≥30 to <40	27 (46.6)
	≥40 to <50	23 (39.7)
	≥50 to <60	7 (12.1)

Clinical experience (years)	<5	3 (5.2)
	≥5 to <10	17 (29.3)
	≥10 to <15	13 (22.4)
	≥15 to <20	13 (22.4)
	≥20 to <30	12 (20.7)

Type of KMD license	General practitioner	30 (51.7)
	Specialist	28 (48.2)

Working institution	KM clinic specialized in pediatric care	29 (50.0)
	General KM clinic	13 (22.4)
	Hospital	16 (27.6)

Number of patients with ISS (monthly average)	<10	27 (46.6)
	≥10 to <30	17 (29.3)
	≥30 to <50	6 (10.3)
	≥50	8 (13.8)

Mean age group of patients with ISS (years)	Infancy (<3)	5 (8.6)
	Preschool (≥3 to <6)	19 (32.8)
	Prepubertal (≥6 to <10)	28 (48.3)
	Adolescence (≥10 to <20)	6 (10.3)

Total		58 (100.0)

KM, Korean medicine; KMD, Korean medicine doctor; ISS, idiopathic short stature.

**Table 2:** Diagnosis pattern of idiopathic short stature in respondents.

Diagnosis pattern		*n* (%)
What indications do you use when ISS treatment? (Duplicate response)	Heights of parents	57 (98.3)
	Height, weight, and growth rate of child	55 (94.8)
	Amount of meal, digestive function	52 (89.7)
	Pattern identification (辨證)	38 (65.5)
	Growth plate test (*X*-ray)	37 (63.8)
	Pulse diagnosis (脈診)	36 (62.1)
	Abdominal diagnosis (腹診)	34 (58.6)
	Tongue diagnosis (舌診)	30 (51.7)
	Growth hormone test (blood test)	13 (22.4)
	Growth plate test (ultrasonography)	3 (5.2)

What accompanied diseases do you check when ISS treatment? (Top 3)	Digestive diseases	53 (91.4)
	Respiratory diseases	33 (56.9)
	Allergic diseases	23 (39.7)
	Underlying disease can cause growth disorder	22 (37.9)
	Precocious puberty	21 (36.2)
	Obesity	12 (20.7)
	Mental illness (i.e. sleep disorder, anxiety)	10 (17.2)

ISS, idiopathic short stature.

**Table 3:** Treatment pattern of idiopathic short stature in respondents.

	Herbal medicine	Acupuncture	Moxibustion	Dry cupping	Physiotherapy	Electroacupuncture	Pharmacopuncture	Chuna
Yes	58 (100)	49 (84.5)	38 (65.5)	26 (44.8)	22 (37.9)	20 (34.5)	20 (34.5)	20 (34.5)

Frequency (n = 49, no response = 9)								
Once a week		31 (63.3)	22 (57.9)	14 (53.8)	14 (63.6)	14 (70.0)	16 (80.0)	16 (80.0)
Twice a week		17 (34.7)	16 (42.1)	11 (42.3)	8 (36.4)	5 (25.0)	3 (15.0)	4 (20.0)
3 times a week		1 (2.0)	0	1 (3.8)	0	1 (5.0)	1 (5.0)	0

Treatment period (n = 58)								
<1 month	2 (3.4)	3 (6.1)	2 (5.2)	1 (3.8)	0	1 (5.0)	0	0
≥1 and <2 months	12 (20.7)	3 (6.1)	3 (7.9)	3 (11.5)	2 (9.1)	2 (10.0)	2 (10.0)	1 (5.0)
≥2 and <3 months	20 (34.5)	10 (20.4)	7 (18.4)	7 (26.9)	3 (13.6)	5 (25.0)	3 (15.0)	4 (20.0)
≥3 and <6 months	16 (27.6)	15 (30.6)	13 (34.2)	7 (26.9)	12 (54.5)	5 (25.0)	6 (30.0)	7 (35.0)
≥6 and <12 months	4 (6.9)	9 (18.4)	6 (15.8)	6 (23.1)	3 (13.6)	5 (25.0)	5 (25.0)	4 (20.0)
≥1 year	4 (6.9)	9 (18.4)	7 (18.4)	2 (7.7)	2 (9.1)	2 (10.0)	4 (20.0)	4 (20.0)

All data are *n* (%).

**Table 4:** Details of interventions for idiopathic short stature.

Intervention		*n* (%)
Purpose of herbal prescription (*n* = 58)	Tonifying the spleen (補脾)	30 (51.7)
	Tonifying the spleen and the kidney (補脾腎)	11 (19.0)
	Tonifying the kidney (補腎)	7 (12.1)
	Tonifying the liver and the kidney (補肝腎)	6 (10.3)
	Others	4 (6.8)

Frequently used herb (*n* = 55, no response = 3)	Acanthopanacis cortex (五加皮)	23 (41.8)
	Astragali Radix (黃芪)	23 (41.8)
	Cervi parvum cornu (鹿茸)	21 (38.2)
	Rehmanniae Radix preparata (熟地黃)	18 (32.7)
	Atractylodis rhizoma alba (白朮)	16 (29.1)
	Dipsaci Radix (續斷)	14 (25.5)
	Angelicae gigantis Radix (當歸)	12 (21.8)
	Ginseng Radix (人蔘)	12 (21.8)
	Achyranthis Radix (牛膝)	9 (16.4)
	Eucommiae cortex (杜仲)	9 (16.4)
	Citri unshius pericarpium (陳皮)	8 (14.5)
	Dioscoreae rhizoma (山藥)	7 (12.7)
	Corni fructus (山茱萸)	6 (10.9)

Frequently used acupuncture points (*n* = 58)	ST36 (zusanli)	48 (82.8)
	GB34 (yanglingquan)	36 (62.1)
	SP6 (sanyinjiao)	32 (55.2)
	EX-LE5 (xiyan)	28 (48.3)
	LI4 (hegu)	26 (44.8)
	BL60 (kunlun)	16 (27.6)
	KI3 (taixi)	15 (25.9)
	KI4 (dazhong)	12 (20.7)
	GB39 (xuanzhong)	11 (19.0)
	GV20 (baihui)	9 (15.5)
	CV12 (zhongwan)	3 (5.2)

**Table 5:** Effects of height growth before and after Korean medicine treatment.

		Before KM treatment	After KM treatment
Boys	Before puberty	4.10 (0.71) cm	6.03 (0.98) cm
	Puberty (rapid growth period)	6.50 (1.29) cm	9.03 (1.56) cm

Girls	Before puberty	4.14 (0.78) cm	5.83 (1.05) cm
	Puberty (rapid growth period)	6.14 (1.24) cm	8.36 (1.71) cm

KM, Korean medicine. All data are in mean (standard deviation).

**Table 6:** Cost of each intervention for idiopathic short stature.

	Herbal medicine (15 days) (*n* = 58)	Acupuncture (*n* = 49)	Moxibustion (*n* = 38)	Dry cupping (*n* = 26)	Physiotherapy (*n* = 22)	Electroacupuncture (*n* = 20)	Pharmacopuncture (*n* = 20)	Chuna (*n* = 20)
>USD9	—	22 (44.9)	32 (84.2)	23 (88.5)	19 (86.4)	7 (35.0)	3 (15.0)	1 (5.0)
≥USD9 and >USD11	—	12 (24.5)	3 (7.9)	1 (3.8)	3 (13.6)	7 (35.0)	3 (15.0)	2 (10.0)
≥USD11 and >USD13	—	5 (10.2)	1 (2.6)	—	—	2 (10.0)	3 (15.0)	1 (5.0)
≥USD13 and >USD15	—	2 (4.1)	—	—	—	—	1 (5.0)	1 (5.0)
≥USD15 and >USD17	—	1 (2.0)	—	—	—	—	7 (35.0)	5 (25.0)
≥USD17 and >USD22	—	7 (14.3)	2 (5.3)	2 (7.7)	—	4 (20.0)	2 (10.0)	8 (40.0)
≥USD22	—	—	—	—	—	—	1 (5.0)	2 (10.0)
≥USD44 and >USD134	3 (5.2)	—	—	—	—	—	—	—
≥USD134 and >USD156	3 (5.2)	—	—	—	—	—	—	—
≥USD156 and >USD178	13 (22.4)	—	—	—	—	—	—	—
≥USD178 and >USD223	15 (25.9)	—	—	—	—	—	—	—
≥USD223 and >USD268	17 (29.3)	—	—	—	—	—	—	—
≥USD268	7 (12.1)	—	—	—	—	—	—	—

USD, United States dollar. It was based on the annual average exchange rate in 2020 from the Korea exchange bank. All data are in *n* (%). Cost of every intervention except herbal medicine were based on 1 visit.

**Table 7:** Opinions on growth treatment in respondents.

Question	Answer	*N* (%)	
		1st rank	Sum of 1^st^–3^rd^ rank
Opinion on Korean-Western medicine collaboration for growth disorder treatment	Korean medicine treatment is more cost-effective than growth hormone.	28 (48.3)	—
	It is best to combine herbal medicine, acupuncture and growth hormone.	22 (37.9)	—
	Health promotion program comprising exercise and diet is more effective in case of ISS without underlying diseases.	8 (13.8)	—

Essential interventions that should be included in health promotion program for pediatric growth	Herbal medicine (decoction)	45 (77.6)	52 (89.7)
	Herbal medicine (products)	4 (6.9)	18 (31.0)
	Diet and lifestyle education	3 (5.2)	31 (53.4)
	Chuna	2 (3.4)	8 (13.8)
	Exercise	2 (3.4)	20 (34.5)
	Acupuncture	1 (1.7)	28 (48.3)
	Pharmacopuncture	1 (1.7)	7 (12.1)
	Cupping	—	4 (6.9)
	Moxibustion	—	4 (6.9)
	Physiotherapy	—	2 (3.4)

Limitation of Korean medicine treatment for pediatric growth	High cost	18 (31.0)	44 (75.9)
	Not covered with health insurance	14 (24.1)	37 (63.8)
	No immediate effect	12 (20.7)	29 (50.0)
	Lack of clinical evidence	7 (12.1)	32 (55.2)
	Lack of publicity	7 (12.1)	32 (55.2)

Appropriate herbal medicine for insurance drugs	Yukmijihwang-tang (六味地黃湯)	25 (43.1)	47 (81.0)
	Sogunjung-tang (小建中湯)	14 (24.1)	43 (74.1)
	Yukgunja-tang (六君子湯)	8 (13.8)	31 (53.4)
	Sipjeondaebo-tang (十全大補湯)	5 (8.6)	28 (48.3)
	Sagunja-tang (四君子湯)	3 (5.2)	15 (25.9)

## Data Availability

The data that support the findings of this study are available from the corresponding author upon reasonable request.

## Abbreviations

EATM: East Asian traditional medicine
GH: Growth hormone
ISS: Idiopathic short stature
KM: Korean medicine
KMD: Korean medicine doctor.
